# Near-cure in patients with Gadolinium deposition disease undergoing intravenous DTPA chelation

This article has been retracted.

**DOI:** 10.3389/ftox.2024.1371131

**Published:** 2024-07-25

**Authors:** Richard C. Semelka, Miguel Ramalho

**Affiliations:** ^1^ Consulting PLLC, Chapel Hill, NC, United States; ^2^ Department of Radiology, Hospital da Luz, Lisbon, Portugal

**Keywords:** Gadolinium, Gadolinium deposition disease, chelation, flare, near-cure

## Abstract

**Purpose:**

To demonstrate and evaluate factors contributing to near-cures in patients with Gadolinium Deposition Disease (GDD) undergoing intravenous (IV) DTPA chelation.

**Methods:**

Patients who had undergone or are currently undergoing DTPA chelation for GDD were included in this report based on their medical records that showed their perceived improvement was at least 80% back to normal. A survey was developed that included factors commonly reported by patients treated in one clinic to determine if these ‘near-cured’ (pre-MRI baseline health) individuals possessed certain factors and lacked others. The anonymized survey was emailed to these individuals by the principal treating physician, the only investigator not blinded to the subjects. This report describes clinical documentation of patient status and their underlying factors in individuals treated by the primary author, and no research was performed. The survey was sent to sixteen individuals; Fourteen patients completed it (10 females; 41.1 ± 11.2 y/o).

**Results:**

The most common factor was the administration of ≤5 lifetime doses of a Gadolinium-Based Contrast Agents (GBCA) (12/14). Unconfounded agents triggering GDD were seen in nine subjects. Most subjects (12/14) initiated chelation in the first year after the causative GBCA, and most (11/14) underwent ≤10 chelations with DTPA. Good healthcare status prior to MRI was observed in 5 subjects. The majority (11/14) described their immune status as strong. Severe physical disability prior to chelation was seen in 1.

**Conclusion:**

Subjects with GDD can experience near-cure with IV DTPA chelation. Factors surveyed that predict near-cure include the start of chelation in the first year, few GBCA administrations, and good health status before MRI with GBCA injection. Nonetheless, a few patients with predictors of less successful outcomes still experienced near-cure.

## Introduction

Gadolinium Deposition Disease (GDD) is a recently described disease that describes a severe persistent reaction to the IV administration of a Gadolinium-Based Contrast Agent (GBCA) (Semelka et al., 2016a; Semelka et al., 2016b; Burke et al., 2016; Semelka et al., 2016c; Semelka and Ramalho, 2021; Semelka and Ramalho, 2023). Other authors have published scientific studies on the entity (Do et al., 2020; Denmark et al., 2022; Jackson et al., 2022). Recently, another group of authors has proposed an alternate designation, Symptoms Associated with Gadolinium Exposure (SAGE), which acknowledges that a reaction to GBCA exists (McDonald et al., 2022; Shahid et al., 2022). SAGE, by its broad definition, should also include acute hypersensitivity reaction (AHR) and nephrogenic systemic fibrosis (NSF) (Semelka and Ramalho, 2023). Nonetheless, there is now broad recognition of the disease process GDD.

Prior reports have described the use of the currently most stable available chelator DTPA (Weinmann et al., 1984; Metal chelates, 2023) for the removal of Gd and have reported on features such as improvement (Semelka et al., 2018) and the increase of Gd removal following chelation compared to pre-chelation (Semelka et al., 2018; Maecker et al., 2020; Maecker et al., 2021; Maecker et al., 2022). No prior report has described whether chelation results in an adequate return to health status before GBCA injection. This report presents patient factors observed in individuals who experienced near-cure of GDD with DTPA chelation therapy.

## Methods

### Patients

This report describes clinical documentation of patient status and underlying factors, and no research was performed. All clinical work and reporting was conducted strictly following the recommendations from the Declaration of Helsinki (Declaration of Helsinki, 2023).

The onset of GDD was considered when symptoms that are consistent with GDD first developed. The principal author asked the patients if, considering all symptoms in total, they considered themselves back to at least 80% of their perceived state of health before GDD. Patients were selected who had either completed chelation or were ongoing chelation by the principal author, who was also directly involved in their care, in whom medical records and subjective perception showed they were at least 80% back baseline health. Individuals who had not improved substantially based on the principal author’s direct assessment were not asked to participate in the survey. Three individuals who did appear substantially improved by the principal author did not take part in the survey as they reported that they did not feel they were 80% back to their former selves.

The primary physician emailed these individuals an anonymized survey to complete (Figure 1). The primary physician was the only investigator aware of their identity.

**FIGURE 1:** Survey: Gadolinium deposition disease near cures.

Sixteen patients who self-reported a return to at least 80% were emailed the survey, and 14 completed it (10 females, 4 males; 41.1 ± 11.2 y/o). All subjects were made aware that the survey was intended for publication. This report does not present a comprehensive list of all subjects seen by the primary physician who may have experienced near-cure but represents individuals who self-report to improve by at least 80% and maintained relatively close contact with the primary physician.

## Results

Tables 1, 2 contain the patients’ survey information.

**TABLE 1:** Recovery from GDD clinical findings.

Subjects	How would you rate your recovery from GDD?	How long are you past your last chelation with DTPA?	How many chelation sessions have you had with DTPA?	How many chelation sessions with other chelator?	Engaged in other forms of detoxification?	How long has it been since you developed GDD?	How soon after GBCA injection did you start chelation?	How many GBCA injections?	Do you know what agent caused GDD?
1	80%–90%	6 months- 1 year	5 to 10	0	no	>2 years	6–12 months	1	MultiHance
2	80%–90%	1–6 months	5 to 10	5 to 10	yes	>2 years	1–2 years	6 to 10	MultiHance
3	90%–95%	>1 year	<5	0	no	>2 years	<3 months	2 to 5	Gadavist and Dotarem
4	90%–95%	1–6 months	>20	0	no	>2 years	1–2 years	>10	Optimark and Gadavist
5	80%–90%	>1 year	5 to 10	0	yes	>2 years	3–6 months	2 to 5	MultiHance
6	80%–90%	6 months–1 year	<5	0	no	1–2 years	6–12 months	2 to 5	Dotarem
7	80%–90%	1–6 months	10 to 20	0	yes	1–2 years	6–12 months	2 to 5	Dotarem
8	80%–90%	6 months–1 year	<5	>20	yes	>2 years	<3 months	2 to 5	Magnevist Unknow
9	90%–95%	1–6 months	5 to 10	0	yes	>2 years	6–12 months	2 to 5	Gadavist
10	80%–90%	1–6 months	<5	0	no	1–6 months	<3 months	2 to 5	MultiHance and Magnevist
11	90%–95%	1–6 months	<5	0	yes	6–12 months	3–6 months	1	Gadavist
12	80%–90%	1–6 months	5 to 10	0	yes	6–12 months	3–6 months	1	Gadavist
13	80%–90%	6 months–1 year	<5	0	yes	6–12 months	6–12 months	1	Dotarem
14	80%–90%	>1 year	<5	0	no	>2 years	<3 months	2 to 5	ProHance and Dotarem

**TABLE 2:** Reasons for obtaining GBCA-enhanced MRI.

Subjects	Before you developed GDD, did you have any of the following	Why was the causative MRI done?	Before GDD, would you describe your immune system as strong?
1	Major accident, or surgery prior to MRI with GBCA	Investigation of minor benign finding, including benign tumor or headache	yes
2	Major accident or surgery prior to MRI with GBCA	Screening for cancer or other disease	yes
3	Autoimmune disease	Screening for cancer or other disease	no
4	None	Investigation of minor benign finding, including benign tumor or headache	yes
5	Major accident or surgery prior to MRI with GBCA	Investigation of major surgery	yes
6	None	Investigation of minor benign finding, including benign tumor or headache (heart)	yes
7	Other	Investigation of minor benign findings, including benign tumors or headache	yes
8	Severe sensitivity to chemicals/drugs. Severe mast cell activation syndrome. EBV or another virus. Major accident or surgery prior to MRI with GBCA	Investigation of major surgery	no
9	MTHFR gene mutation	Investigation of minor benign finding, including benign tumor or headache	yes
10	EBV or another virus	None of the above	yes
11	Lyme	Investigation of major autoimmune or autoinflammatory disease	yes
12	Severe sensitivity to chemicals/drugs, Major accident, or surgery prior to M MRI Ri with GBCA, High potency antibiotics prior to MRI with GBCA	Screening for cancer or other disease	yes
13	Other	Investigation of minor benign finding (back pain)	yes
14	Autoimmune disease, severe sensitivity to chemicals/drug	Investigation of major surgery	no

Most subjects (8/14) received two to five GBCA doses, and four received only 1 GBCA.

Twelve subjects initiated chelation sessions in the first year after the causative administration of a GBCA. Four subjects initiated chelation <3 months after the triggering GBCA, three between 3–6 months, five between 6–12 months, and two between 1–2 years.

Unconfounded agents triggering GDD were seen in nine subjects (MultiHance in 3, Dotarem in 3, and Gadavist in 3).

Two subjects underwent previous chelation with other agents without satisfactory results.

Eleven subjects underwent ≤10 chelation sessions with DTPA.

Good healthcare status prior to MRI was observed in five subjects. Eight subjects engaged in other forms of detoxification. The majority (11/14) described their immune status as strong. Severe physical disability prior to chelation was seen in one.

## Discussion

The primary observation in this report is that subjects with GDD can experience near-cure of the disease with IV DTPA chelation, including those with >5 GBCA doses. This is important, as individuals with other similar diseases, such as fibromyalgia or stiff person disease, can be managed with medical care but not treated to near-cure (Varrassi et al., 2023). The second important observation is that most subjects who experience near-cure began chelation <12 months after the development of GDD.

Not surprisingly, most near-cures occur in individuals who received few lifetime GBCA administrations. Possible explanations include: 1) the total body Gd burden is relatively low, hence easier to remove the bulk of retained heavy metal, and 2) in individuals who have received multiple GBCA injections, each subsequent GBCA injection makes the condition worse, hence the severity of disease in generally worse in those who received multiple GBCAs (Semelka and Ramalho, 2023). It is also an expected outcome that individuals who were in general good health prior to GBCA injections (for example, one individual who received multiple GBCA injections to follow a small intracranial meningioma) should also be more likely to return to good health with DTPA chelation.

In the conception phase of this report, the authors had anticipated reporting on cures of GDD from the success of DTPA chelation therapy. Following 6 years of clinical experience and patient follow-up, it has become apparent that a complete cure for this disease may not occur with any frequency. Instead, individuals experience near-cure. Although this appears disappointing on the surface, the reality is that this circumstance is observed in many diseases where the mechanism is invasion by some external pathogen. Therefore, GDD near-cure appears analogous to entities such as Herpes or Varicella infection. The individual is effectively near-cured but still harbors elements of the pathogen, which may arise and become symptomatic again at a future date, but these recurrences are generally very manageable. This is likely the case with GDD, in which at moments of various kinds of stress, such as psychological, injury, or hormonal change, symptoms may at least transiently recur. This persistence of the prospect of recurrence is likely not dire but rather a somewhat common circumstance that individuals deal with from several conditions.

Most patients underwent ≤10 chelations. A critical point also worth mentioning is that in individuals who experience near-cure, perseverance in obtaining chelations every 1–4 weeks is essential, regardless of whether the Flares are severe. The results of our clinical experience suggest that our IV DTPA regimen is now sufficiently mature, and at this point, actual scientific investigations, such as Randomized Control Trials (RCTs), can be meaningfully performed.

Optimistic findings in our report for the larger population of sufferers are that even individuals who received multiple injections or who were significantly disabled at the time of chelation start may also achieve near-cure from the disease. Two such individuals described themselves as > 95% recovered, underwent a considerable number of chelations, and severe flare reactions complicated their treatment course, especially in the early stages. However, it must be noted that they did not get concurrent steroid administration for the majority or all their chelations, which is essential to dampen the Flare reaction (Semelka et al., 2018; Maecker et al., 2021; Semelka et al., 2021; Semelka and Ramalho, 2023). The approach we have employed for at least 2 years is to start chelation at a lower level of volume (2.5 mL of chelator, compared to the standard volume in the marketed product of 5 mL) of just Zn-DTPA combined with 125 mg iv solumedrol with a subsequent oral steroid and antihistamine taper. The volume of the chelator is increased to 1 vial Ca-DTPA day 1 and 1 vial ZnDTPA day 2, and the amount of steroid decreased, with further chelation, based on the individual’s tolerance to Flare reactions.

Limitations of this report include that this is a descriptive work documenting clinical experience and not a controlled research study. However, it has become appreciated in medical literature that real-world experience is a powerful method to evaluate the success of various treatments (Semelka et al., 2016a; Chodankar, 2021). Nonetheless, an RCT comparison with alternative treatment methods, most appropriately with potent Gd chelators such as HOPO but including no treatment at all, has yet to be studied, which will be critical. The principal explanation is that treatment for GDD is still in its early stages, and the authors report their clinical experience with a treatment regimen that makes the most empirical sense of available treatments. If a substance is embedded in the body and is making the individual unwell, the primary treatment should be the removal of that substance (Kim et al., 2018; Maecker et al., 2021; Semelka and Ramalho, 2023). Alternative science-supported treatments have not been reported in the literature, so alternative therapies are not used in the treating clinic for patient care.

Nonetheless, patients have reported on patient support websites that they have experienced cures with other approaches, including no specific treatment. In our opinion, it is not rare that following just a one-lifetime dose of GBCA injection, recovery without specific targeted therapy beyond support and diet does occur, as described by sufferers in online forums/support groups and direct communication with the principal author. We postulate that what is occurring in these individuals is that their immune system eventually resets to baseline function. In fact, as we perform IV chelation DTPA, we aim to pause chelation when the individual is 80%–85% improved to allow for the same effect: self-calming of the immune system despite the persistent presence of at least trace Gd. The advantage of chelation over no Gd removal and pure immune system self-calming is that the effect of chelation results in much less Gd remaining in the body, hence a much smaller quantity to serve as the impetus to inflame the body in the future from either spontaneous flare or from further GBCA injection. Through discussion with several sufferers, most of whom received just one-lifetime GBCA injection, who opted for no chelation treatment, it appears that near-cure without specific treatment takes approximately 2 years. Near-cure without chelation following multiple GBCA injections appears exceedingly exceptional but can happen. Based on this 2-year timeline, we also use this to explain to individuals who have undergone chelation therapy that when they suspend further chelation at their self-perception of 80% recovery, further spontaneous recovery to 95% or greater will eventually take approximately 1–2 years. The beneficial difference for individuals who have undergone chelation compared to those who have not is that their starting point for further recovery is at a much higher level of functioning and symptom relief than those who undergo spontaneous recovery alone, where their status is often at 20%–30% of their former self, rather than 80%, as in the post-chelation group.

A further limitation of this report is that it was not designed to determine the percentage of individuals undergoing DTPA chelation therapy going on to near-cure. The explanations are several: many patients who come to the primary author’s clinic travel from some distance, and our standard practice is to facilitate the patient receiving further chelation care after their second chelation at our center, at a practice closer to where they live. The primary reasons are cost and convenience. Many individuals opt to stop chelation at a lower level of their perception of return to pre-GDD status; 70% is a level many describe, and the primary explanations appear to be the cost of treatment and convenience. Thirdly, some individuals do not continue to communicate with their treating centers, and a primary explanation is that when they are feeling better, they prefer to avoid the subject of GDD. Fourthly, individuals being chelated at other centers for further care may receive different treatment types. Hence, their status may not reflect the effect of DTPA chelation. Considering these limitations, we believe that most individuals experience substantial benefits from DTPA chelation for their care, and the primary impediment to obtaining sufficient chelation to achieve 80% recovery appears to be the cost of the treatment. In general terms, though, the findings from our clinic experience should provide hope to patients that the disease is highly treatable.

It should be emphasized that this population of patients reported herein does not represent the total number of patients who have achieved near-cure or will achieve near-cure; many patients have started chelation whose trajectory will likely accomplish that goal. A final point is that even those who have received multiple GBCA injections will still show substantial improvement with chelation, even if they do not achieve the goal of 80% recovery. A few patients were requested to enter this report because of their considerable improvement. However, they declined because although their recovery was substantial, they felt they did not hit the mark of 80% recovery.

Since GDD is often an “invisible disease” defined almost entirely by symptoms, doubts remain even to this day as to whether it is a real clinical condition (McNamara and Rahmani, 2018; Harvey et al., 2020; Layne et al., 2020; van der Molen et al., 2024). The most crucial evidence arguing in favor of its existence is the findings of causation from GBCA administration: i) in the present and prior reports, patients described that GDD onset occurred shortly after administration of a GBCA (Semelka et al., 2016b; Burke et al., 2016; Semelka et al., 2016c; Semelka and Ramalho, 2021), ii) Gd has been demonstrated in the urine of GDD patients some months after GBCA injection (Semelka et al., 2016b; Burke et al., 2016; Semelka et al., 2016c; Semelka and Ramalho, 2021), iii) removal of Gd with DTPA chelation has been shown on pre- and post-DTPA chelation 24-h urine samples (Semelka et al., 2016c; Semelka et al., 2018; Maecker et al., 2020; Maecker et al., 2021; Maecker et al., 2022), iv) patients have shown improved symptoms following chelation (Semelka et al., 2018), and finally v) with continued chelation, individuals can experience near-cure (this present report). In contrast, with Nephrogenic Systemic Fibrosis, this level of proof was never attained, as removal of the purported causative agent of disease was never shown, nor, more importantly, with continued removal of the causative agent near-cure achieved.

In summary, subjects with GDD can experience near-cure with IV DTPA chelation. The most likely to achieve this are those with few GBCA injections, those who start chelation in the first year, and those without significant pre-existent disease of various causes. This emphasizes the imperative for healthcare workers to recognize GDD as soon as it arises, such as after the first GBCA injection, as these individuals are the most likely to recover completely. More research is needed.

## Data Availability

The raw data supporting the conclusions of this article will be made available by the authors, without undue reservation.
